This article has been retracted.

# Effects of microRNA-101-3p on predicting pediatric acute respiratory distress syndrome and its role in human alveolar epithelial cell

**DOI:** 10.1080/21655979.2022.2070583

**Published:** 2022-05-04

**Authors:** Fang Yin, Qi Li, Min Cao, Yaqin Duan, Liu Zhao, Lumin Gan, Zili Cai

**Affiliations:** a Child Health Development Center, Hunan Children′s Hospital, Changsha China; b Rehabilitation Center, Hunan Children′s Hospital, Changsha China; c Children’s Research Institute, Hunan Children′s Hospital, Changsha China; d Department of Infection, Hunan Children′s Hospital, Changsha China

**Keywords:** miR-101-3p, PARDS, inflammation, diagnosis, sox9

## Abstract

Pediatric acute respiratory distress syndrome (PARDS) is a severe form of respiratory failure associated with high mortality among children. The objective of this study is reported to explore the clinical function and molecular roles of microRNA-101-3p (miR-101-3p) in PARDS. The levels of miR-101-3p and mRNA levels of SRY-related high-mobility group box 9 (Sox9) were measured by quantitative reverse transcription polymerase chain reaction (RT-qPCR). Additionally, the diagnostic role of miR-101-3p was identified by using the Receiver operating characteristic (ROC) curve. The cell proliferation and apoptosis were examined through Cell Counting Kit-8 (CCK-8) assay and flow cytometry. To detect inflammation in cells, enzyme-linked immunosorbent assays (ELISA) were performed. The target gene of miR-101-3p was confirmed through data obtained from the luciferase activity. In patients with PARDS, miR-101-3p expression was decreased. Moderate and severe PARDS patients had lower levels of miR-101-3p than mild PARDS patients. The inflammatory progression was related to the aberrant expression of miR-101-3p in all PARDS children. MiR-101-3p was highly predictive for the detection of children with PARDS. In addition, miR-101-3p might protect A549 cells from abnormal proliferation, apoptosis, and inflammation caused by lipopolysaccharide (LPS). Sox9 might be a target gene of miR-101-3p and increased mRNA expression of Sox9 in LPS-treated A549 cells was inhibited by overexpression of miR-101-3p. Ultimately, this study suggested that reduced expression of miR-101-3p plays a role in PARDS, providing a novel angle to study the disease.

## Highlights

- The expression of miR-101-3p was decreased in patients with PARDS.
- Among LPS-treated A549 cells, miR-101-3p played an important role.
- MiR-101-3p might be a biomarker for screening PARDS patients.
- Sox9 was directly targeted by miR-101-3p.

## Introduction

Acute respiratory distress syndrome (ARDS) is a severe illness with complex clinical symptoms [1]. The symptoms of ARDS include pulmonary edema, respiratory insufficiency, and hypoxemia caused by noncardiogenic reasons (such as infection, shock, trauma, or high-risk surgery) [2]. The diagnosis of ARDS cannot be confirmed or ruled out with a single test. Pediatric ARDS (PARDS) occurs across the entire pediatric age group [3]. Despite its low incidence, PARDS has a high mortality rate of 34% [4]. Additionally, neurologic failures, such as non-traumatic brain damage and multisystem organ dysfunction become the primary reasons for mortality during the PARDS progression [5]. Approximately 63% of those with PARDS have co-morbidities at the time of diagnosis and have preexisting co-morbidities, including lung disorders, prematurity, chronic respiratory support, congenital heart disease, immune suppression, and cancer [6]. Children with PARDS are often hospitalized and require mechanical ventilation, which further adds to the burden placed on families [7]. Investigation of PARDS development is therefore imperative.

Recently, several publications have been published in ARDS that focus on miRNAs. Several publications on miRNAs have been published in the field of ARDS. The levels of serum microRNA-127 (miR-127) in the ARDS patients are significantly raised and the predictive role of miR-127 is also revealed by Lin et al, which elucidated that differentially expressed miRNA has the potential to be a biomarker [8]. ARDS is a syndrome stimulated by damaged alveolar epithelial cells and inflammation [9]. Lipopolysaccharide (LPS) treatment of lung alveolar epithelial cells can lead to acute cell injury, which is the main characteristic of ARDS [10]. In a study by Hou et al., ARDS cell models were constructed using A549 cells, and miR-297 was demonstrated to be relevant to cell proliferation and inflammation [11]. Another study provides the significant effects of miR-296-5p on neonatal ARDS by transfecting lentivirus encoding miR-296-5p into A549 cells [12].

During the last few decades, the expression and influence of miR-101-3p have gained significant attention. MiR-101-3p is implicated in the regulation of chondrocyte inflammation in osteoarthritis, indicating that miR-101-3p is related to the inflammatory response [13]. In colorectal cancer, miR-101-3p plays a role in radiation resistance. Additionally, the decrease in miR-101-3p expression was confirmed in a model of acute lung injury induced by bleomycin, which is a predisposition to the development of ARDS. These previous investigations imply that miR-101-3p may play a role in the progress of PARDS. SRY-related high-mobility group box 9 (Sox9) is widely researched recently, which arises our interest. For instance, Sox9 plays an important role in lung function recovery in acute lung injury [14]. In addition, inflammation is a major cause of ARDS, and tumor necrosis factor alpha (TNF-α), interleukin-6 (IL-6), and interleukin-17 (IL-17) are three common proinflammatory factors [15,16]. Thus, studying inflammation is crucial in PARDS.

Considering these, we hypothesized that the expression of miR-101-3p might be influenced by PARDS and the change of miR-101-3p expression was a risk of PARDS. It was hypothesized that miR-101-3p affected the proliferation, apoptosis, and inflammation in LPS-induced A549 cells and Sox9 was a target of miR-101-3p in PARDS. This study aimed to test the roles and values of miR-101-3p in PARDS and to identify a biomarker for this disease. As part of our analysis, we collected serum samples from all participants with PARDS and evaluated the levels of miR-101-3p in their serums. The Receiver Operating Characteristic (ROC) curves demonstrated the clinical diagnosis of miR-101-3p. Moreover, the effects of miR-101-3p on LPS-triggered A549 cell models were investigated to discover the significance of miR-101-3p on PARDS.

## Materials and methods

### Patients and sample collection

A total of 82 children with PARDS admitted to the Hunan Children′s Hospital were selected as research subjects and 77 healthy children were selected as the control group. We verified the PARDS patients using consensus recommendations published in 2015 and we excluded patients with acute hypoxemia unique to the perinatal period or with other congenital abnormalities [3]. All the included patients were in the acute phase, that is, the onset of symptoms for all the patients was less than 3 days. According to the Berlin Definition, the eligible PARDS subjects were divided into three groups, mild, moderate, and severe [17]. The healthy children did not have infectious disease or use immunosuppressant in the past month. The Ethics Committee of Hunan Children’s Hospital approved the design of this study[Approval number: 20,180,031]. The legal guardians of all subjects gave informed consent and signed the consent form.

### Cell model construction and transfection

In order to establish the model of PARDS in vitro, human alveolar epithelial cell line A549 was obtained from the cell bank (Shanghai, China). These cells were fostered in the Dulbecco’s modified eagle’s medium containing 10% FBS. Cells with 80% confluence were treated with 1 g/ml LPS for 24 hours [18].

The miR-101-3p mimics, miR-101-3p inhibitors, and miRNA negative controls (miR-NC) were purchased from Genepharm (Shanghai, China). Lipofectamine 3000 (ThermoFisher, USA) was the main reagent used in the transfection [19]. After 48 hours, all transfected cells were harvested.

### Identification of miR-101-3p expression

About 3 ml peripheral blood were collected from PARDS patients and healthy children. A total RNA blood kit (ThermoFisher, USA) was used to extract total RNA [20]. The concentration and purity of RNA have been detected by measuring their optical density (OD)_260_ and OD_280_ [21]. A complementary DNA (cDNA) synthesis kit (NovaBio, Shanghai, China) was used to obtain single sequences of cDNA [22]. The expression of miR-101-3p was measured by a miRNA qPCR mix from Sangon Biotech (Shanghai, China) [23]. The relative levels of miR-101-3p were normalized by the expression of U6 using the 2-DeltaDeltaCT method [24].

### Cell proliferation assay

The Cell Counting Kit-8 (CCK-8) from the absin (Shanghai, China) was applied to measure cell proliferation [25]. A density of 5 × 10^3^ A549 cells was seeded into each well of a 96-well plate. The plate was incubated in a constant temperature incubator for 24 hours. 10 µl CCK-8 reagent was mixed with cells in each well and then, the proliferation of cells was measured with a microplate at wavelength 450 nm after 48-hour of incubation.

### Cell apoptosis assay

By combining logarithmic growth cells with the binding buffer, a single-cell suspension was prepared. The cell suspension of 100 µl was added to the tube and mixed with 5 µl of Annexin V-EGFP. The experimental cells were incubated in the dark for 5 minutes. Then, 10 µl of the PI solution was added for staining. The flow cytometry kit for detecting apoptotic cell was from Yeason (Shanghai, China) [26]. The flow cytometry examination was completed within one hour.

### Detection of inflammatory mediators

The inflammatory responsesin patients and human alveolar epithelial A549 cells were reflected by the concentration of TNF-а, IL-6, and IL-17. The levels of TNF-α, IL-17, and IL-6 in cell supernatant were measured through Enzyme-linked immunosorbent assay (ELISA) kits based on the recommended procedures (mlbio, Shanghai, China) [27].

### Luciferase report assay

The presence of correlation among Sox9 and miR-101-3p was examined by luciferase assay. The pmirGLO vector was used as the carrier. Both wild type (WT) and mutation type (MUT) Sox9 were obtained by cloning them into pmirGLO to construct WT-Sox9 and MUT-Sox9 vectors. The miR-101-3p mimic, miR-101-3p inhibitor, and miR-NC were transfected into cells with the previous carriers into cells. The luciferase activity was evaluated by a luciferase assay kit (Beyotime, Beijing, China) on a multiscan spectrum [28].

### Statistical analysis

The experimental values were calculated on SPSS and GraphPad software and recorded as number or mean ± SD. A Chi-square test was employed to compare the classification variables, such as gender, etc. Additionally, the continuous variables of the two groups were estimated with the help of a t-test. The differences among three or more groups were confirmed by one-way ANOVA (analysis of variance). We used the multiple linear regression analysis to determine whether miR-101-3p was relevant to inflammation in PARDS. ROC curves were used to demonstrate the diagnostic values, specificity, and sensitivity of miR-101-3p.

## Results

Our aim in this study was to analyze miR-101-3p’s roles in PARDS, and we hypothesized that miR-101-3p might be associated with PARDS. We assessed the expression of miR-101-3p in PARDS patients and evaluated its diagnostic potential. Additionally, miR-101-3p has been shown to influence the proliferation, apoptosis, and inflammation of A549 cells caused by LPS. Furthermore, the direct target of miR-101-3p has been identified.

### Basic clinical information of each individual

We examined the differences between healthy people and PARDS patients. The mean age of PARDS patients was found to be 3.70 ± 2.0 years old. A total of 32 women and 50 men constituted the ARDS group. Age and gender comparisons between the healthy group and PARDS patients did not reach statistical significance (Table 1, *P* > 0.05). In addition, the concentrations of IL-17, IL-6, and TNF-α were higher in the serum of PARDS patients than in the serum of healthy participants (Table 1, *P* < 0.001).

**Table 1.** Basic clinical data of participants

	Participants		
Indicators	Healthy individuals (n = 77)	PARDS patients (n = 82)	*P* value
Gender (women/men)	36/41	32/50	0.325
Age (years)	3.91 ± 2.01	3.70 ± 2.0	0.514
TNF-α (pg/ml)	18.29 ± 0.26	32.78 ± 4.77	< 0.001
IL-6 (pg/ml)	12.43 ± 3.33	18.61 ± 4.34	< 0.001
IL-17 (pg/ml)	105.65 ± 24.45	201.06 ± 29.19	< 0.001

Annotation: PARDS: pediatric acute respiratory distress syndrome; TNF-α, tumor necrosis factor -alpha; IL-6, interleukin-6; IL-1β; IL-17: interleukin-17. Data are expressed as n or mean ± standard deviation.

### Relationship between miR-101-3p expression levels and inflammatory cytokines in PARDS children

As shown in Figure 1a, the serum expression of miR-101-3p was decreased in the PARDS group in comparison to the healthy group (*P* < 0.001), indicating that PARDS might contribute to the dynamic changes in miR-101-3p expression. Furthermore, we assessed the expression of miR-101-3p in 37 patients with mild PARDS, 29 patients with moderate PARDS, and 17 patients with severe PARDS. As shown in Figure 1b, the expression of miR-101-3p was significantly reduced in all subgroups of PARDS when compared with healthy children (*P* < 0.001). Additionally, compared to mild PARDS patients, miR-101-3p expression was decreased in the moderate group and the severe group, respectively (Figure 1b, *p* < 0.001).

**Figure 1.** The expression of miR-101-3p in PARDS patients. **A**. The low expression of miR-101-3p in children with PARDS. **B**. The expression of miR-101-3p in the mild, moderate, and severe PARDS patients. ***P < 0.001, compared with healthy individuals, ###*P* < 0.001, compared with mild group.

All PARDS patients were further examined for associations between miR-101-3p and inflammatory items. As shown in Table 2, the miR-101-3p expression levels were related to the concentration of TNF-α, IL-6, and IL-17, suggesting miR-101-3p might influence the inflammatory condition in PARDS patients (*P* < 0.01).

**Table 2.** Multiple linear regression analysis on variables associated with miR-101-3p

Characteristics	Coefficient	Standard error	t	*P-value*
TNF-α (pg/ml)	−0.006	0.002	−3.052	0.003
IL-6 (pg/ml)	−0.010	0.002	−5.839	<0.001
IL-17 (pg/ml)	0.002	0.000	−6.497	<0.001

Annotation: TNF-α, tumor necrosis factor -alpha; IL-6, interleukin-6; IL-1β; IL-17: interleukin-17.

### The sensitivity and specificity of miR-101-3p in assessing PARDS patients

Further test of the predictive significance of miR-101-3p was performed on PARDS patients. As depicted in Figure 2, an area under the curve (AUC) of 0.939 interpreted the indicative possibility of miR-101-3p. The high accuracy of miR-101-3p was further demonstrated by a sensitivity of 90.2% and a specificity of 85.7% (Figure 2).

**Figure 2.** The AUC of miR-101-3p was 0.939 with a sensitivity of 90.2% and a specificity of 85.7%.

### Importance of miR-101-3p on cell models

To examine the effects of miR-101-3p, A549 cells were constructed and transfected with artificial miR-101-3p sequences. In comparison with control cells, the expression of miR-101-3p was diminished in LPS-induced cells (Figure 3a, *p* < 0.001). The expression of MiR-101-3p was improved in the miR-101-3p mimic group and inhibited in the miR-101-3p inhibitor group compared with the LPS group, predicting the success of artificial transfection (Figure 3a, p < 0.01).

**Figure 3.** The role of miR-101-3p in LPS-evoked cell models. **A**. LPS inhibited miR-101-3p expression, but transfection altered miR-101-3p expression. **B** The findings of CCK-8 on A549 cells showed overexpression of miR-101-3p restricted the influence of LPS and interference of miR-101-3p accelerated the effects of LPS. **C** The beneficial effects of miR-101-3p on cell apoptosis. **D** The inhibitory effect of miR-101-3p on the inflammatory biomolecules in A549 cells. ***P < 0.001, compared with the control cells, #*P* < 0.05, ##*P* < 0.01, ###*P* < 0.001, compared with the LPS group.

As determined by the CCK-8 and flow cytometry assays, LPS suppresses cell proliferation and promoted apoptosis, whereas the augmented miR-101-3p expression mitigated these impacts and the suppressed miR-101-3p expression increases the damaging effects of LPS (Figure 3b-c, *P* < 0.01). Amplification of miR-101-3p slowed down the augmented inflammatory response of LPS-treated cells, and intervention of miR-101-3p expression exacerbated the influence of LPS (Figure 3d, p < 0.05).

### Sox9 was a possible target gene of miR-101-3p

The direct target of miR-101-3p was predicted by bioinformatics. The putative sites between miR-101-3p and Sox9 were shown in Figure 4a. The target connection between Sox9 and miR-101-3p was certified by the luciferase report, which elucidated that miR-101-3p mimics reduced the activities and miR-101-3p inhibitors suppressed the activities in the WT-Sox9 group (Figure 4b, *p* < 0.001). In the LPS group, the relative quantitation of Sox9 was boosted but miR-101-3p overexpression mitigated Sox 9 expression and miR-101-3p underexpression elevated Sox 9 expression. (Figure 4c, *p* < 0.01).

**Figure 4.** Sox9 is a target gene of miR-101-3p. **A** Visualization of the binding sites between Sox9 and miR-101-3p. **B** The luciferase activity was decreased in the miR-101-3p mimic subgroup and increased in the miR-101-3p inhibitor subgroup in WT-Sox9 group. **C** Sox9 mRNA expression was increased in the LPS group, which was compounded by the shift in miR-101-3p expression in A549 cell models. ***P < 0.001, compared with the control cells, ##*P* < 0.01, ###*P* < 0.001, compared with the LPS group.

## Discussion

ARDS is a form of respiratory dyspnea, characterized by intractable hypoxemia and progressive dyspnea [29]. ARDS has a relatively high mortality rate in children, but there are no reliable indicators for estimating the severity of the disease [4]. Therefore, finding PARDS-related indexes has great clinical significance. The clinical pathology of ARDS is primarily characterized by an inflammatory response In the early stage of ARDS, cells in alveoli release a large number of inflammatory indicators, such as TNF-α, that aggravate the inflammatory reaction process and induce lung tissue damage [30]. In the process of inflammatory reaction, IL-17 is also an important inflammatory factor, and its overexpression can cause tissue and cell damage [31]. IL-17 also plays a role in the inflammatory reactions of the lungs [32].

In this study, the expression level of serum miR-101-3p in PARDS children was significantly lower than that of healthy children. The reduction of miR-101-3p expression was accompanied by the severity of PARDS, suggesting that miR-101-3p was related to the severity of ARDS. MiR-101-3p is significantly decreased in patients with idiopathic pulmonary fibrosis and its change is associated with forced vital capacity, which provides evidence that miR-101-3p is important for lung function [33]. The abnormal expression of miR-101-3p is also found in the development of idiopathic condylar resorption [34]. In acute lung injury, the expression of miR-101-3p is diminished in the bleomycin-induced mice models, which further indicates miR-101-3p participates in the development of lung diseases [14]. All these researches provides that PARDS may lead to the change of miR-101-3p expression. Also, the associations of miR-101-3p and inflammation were also validated, that is, the expression of miR-101-3p was closely correlated with the serum content of TNF-а, IL-6, and IL-17, thus suggesting that miR-101-3p impacted inflammation in PARDS. The overexpression of miR-101-3p inhibits the expression of IL-6 and TNF-а in an article about syphilis, which explains the link between miR-101-3p and inflammation [35]. More importantly, the ROC results showed miR-101-3p had a high possibility of predicting PARDS patients from healthy children with a high degree of accuracy. Previous studies also reveal the diagnostic probability of miRNAs in adults with ARDS. A combination of serum miR-92a and miR-146a can improve the diagnostic sensitivity and specificity of the identification method of ultrasound [36]. According to Parzibut et al., seven miRNAs have altered expressions, indicating they could discriminate ARDS patients from healthy individuals [37]. As an alternative diagnostic factor in PARDS, miR-101-3p could also be used as compared to many miRNAs previously studied.

The assays about A549 cells provided further insight into miR-101-3p on LPS-induced cell models. Increased levels of miR-101-3p ameliorated the inhibition of cell proliferation caused by LPS. In addition, the elevated miR-101-3p expression alleviated the boosted cell apoptosis induced by LPS, elucidating miR-101-3p might be a protective marker in the progression of PARDS. The influence of miRNAs in LPS-evoked alveolar cell models has been reported in several publications. For example, overexpression of miR-122-5p modulates the bioactivities of A549 cells which are damaged by LPS [38]. In this study, we also detected the function of miR-101-3p on inflammation, which was induced by LPS and attenuated by high levels of miR-101-3p, suggesting that miR-101-3p had a protective effect on inflammation. Moreover, miR-101-3p is identified as a biomarker in the negative feedback regulation of inflammation in systemic lupus erythematosus [39]. The inhibitory influence of miR-101-3p on the inflammation in rat models of rheumatoid arthritis is also verified [40]. This previous evidence also certifies our findings of miR-101-3p on inflammation.

Further analysis of miR-101-3p was also performed to understand its mechanistic role in PARDS. Sox9 was a target of miR-101-3p in the present study. Cui et al. demonstrate that miR-101-3p and Sox9 have a targeted relationship in non-small cell lung cancer [41]. Furthermore, our findings revealed that LPS increased the expression of Sox9 mRNA, while overexpression of miR-101-3p alleviated this trend, suggesting that miR-101-3p suppresses Sox9 expression. Roles of Sox9 in lung development and function are widely reported [42,43]. In idiopathic pulmonary fibrosis, Sox9 participates in the migration and survival of fibroblasts [44]. Several studies reveal the underlying mechanism of ARDS by conducting in vivo mouse model and an in vitro cell model [45,46]. Compared to these publications, we examined not only the effects of miR-338-3p in A549 cells caused by LPS, but also the diagnostic role of miR-338-3p for PARDS patients.

## Conclusion

Based on the studies, it was found that the expression of miR-101-3p was declined among patients in the condition of mild, moderate, and severe PARDS. Further, in all PARDS patients, the expression of miR-101-3p was correlated with inflammatory mediators. Hence, it was noticed that the expression of miR-101-3p might distinguish PARDS patients from the healthy children group. MiR-101-3p also influenced cell proliferation, apoptosis, and inflammation in response to LPS. Moreover, our results suggest that Sox9 might be a target of miR-101-3p and miR-101-3p inhibited the mRNA expression of Sox9 in LPS-treated cells.
